The article "Adsorption of Malachite Green (MG) as a Cationic Dye on Amberlyst 15, an Ion-Exchange Resin" was published in 2022. Journal: J Environ Public Health.

# Adsorption of Malachite Green (MG) as a Cationic Dye on Amberlyst 15, an Ion-Exchange Resin

**DOI:** 10.1155/2022/4593835

**Published:** 2022-03-21

**Authors:** Amineh Nandoost, Nader Bahramifar, Ali Akbar Moghadamnia, Sohrab Kazemi

**Affiliations:** ^1^Department of Pharmacology, Babol University of Medical Science, Babol, Iran; ^2^Department of Environmental Sciences, Faculty of Natural Resources and Marine Sciences, Tarbiat Modares University, Noor, Iran; ^3^Cellular and Molecular Biology Research Center, Health Research Center, Babol University of Medical Sciences, Babol, Iran

## Abstract

Crystals of malachite green (MG), being water-soluble, are effective agents applied to combat fungal and parasitic infections in fish. This study was conducted to evaluate the adsorption of MG as a cationic dye by polymeric resin Amberlyst 15. Changes in several parameters were observed, including the concentration of MG, pH, the adsorption rate and extent, and the temperature that might all affect the efficiency of adsorption. The adsorption method was described well by both the Redlich–Peterson and Langmuir isotherms with *R*^2^ of 0.9933 and 0.9880, respectively. The kinetic information is consistent with the Freundlich isotherm model and pseudo-2nd-order kinetics model. Analysis of malachite green was executed by HPLC containing a Eurospher 100-5 C18 (25 cm × 4.5 mm, size of particle 5 *μ*m) column, UV detector was set at 618 nm, and 125 mM ammonium acetate was adapted to pH 4.5 with formic acid-acetonitrile (45 : 55, v/v) as the moving phase. The limit of the discovery factor was 0.02 *μ*gL. The negative value of Δ*G*° reveals the spontaneity of the absorption method. The positive value of Δ*S*° (333.1253 J/K mol) gives back randomness at the solid-liquid interface of sorption. The required adsorbent concentration was calculated for removing MG up to an extraction efficiency of 98.27% after 240 minutes.

## 1. Introduction

Population growth and followed industrial activities have been causing environmental problems over the past few decades. Many human industrial activities cause undesirable changes in water quality. Industrial processes usually generate waste materials that if not disposed of properly according to standard conditions of waste disposal, may be harmful to human health [1]. Disposal of dyes in factory-made liquids into drinking water is a prominent issue because in several places such materials are of high defiance to chemical, biological, or photochemical depravity [2, 3]. Dyes are utilized in abundance in many industrial productions, containing textile, leather, cosmetics, cardboard, printing, pharmaceuticals, treated compounds, edible material, etc. [3]. The mentioned dye, malachite green (MG), as a cationic dye, is a tri-phenyl methane dye with the formula C_52_H_54_N_4_O_12_ [1, 4, 5] as well as a fungicide dye that is environmentally stable and as a matter of fact poisonous to a large scale of mundane animals and animals living in water [3]. The presence of organic dyes in the aquatic environment is a serious global trouble because of the dangerous negative consequences on the quality of ecosystems. This dye may be considered a carcinogenic agent, as it can exert its toxic effects on human liver cells, which induces tumor formation [6].

The article "Adsorption of Malachite Green (MG) as a Cationic Dye on Amberlyst 15, an Ion-Exchange Resin" was published in 2022. Journal: J Environ Public Health.

Nevertheless, MG is still being used because of its relative inexpensiveness and good efficacy in blockage and treatment of outside parasitic and fungal contamination [4, 5]. Finding a method for removing MG from aqueous solutions has been of much interest to researchers. Some adsorbent materials such as beech sawdust, rice straw, and orange peel have been introduced as new resources for removal techniques [6–8]. Dhodapkar et al. used bentonite to eliminate MG out of aqueous solution [9]. Dos Reis et al. isolated MG from aqueous solution by adsorption on Amberlite XAD-4 and XAD-2 resins [2].

This study was conducted to investigate the adsorbing capability of Amberlyst 15 (a polymeric resin) for usage in MG-contaminated specimens. The method of UV/V spectrophotometry was used to assay MG [10]. It is largely applied because of its simple function, affordability, and unique properties such as environmental compatibility, nontoxicity, reusability, noncorrosiveness, chemical and physical stability, noticeable precision, and good selectivity and sensitivity [11, 12]. The role of pH, temperature, and concentration of Amberlyst 15 and MG has been investigated [11, 12]. Amberlyst 15 can be produced via the catalytic reaction of methanol (MeOH) and isobutylene (IB4) in the liquid phase using an ion-exchange resin. The object of this study was to assess optimal conditions to obtain the maximum removal effect of MG from aqueous solutions and interpretation of experimental results by comparing them.

## 2. Experimental

### 2.1. Apparatus

An HPLC device made by Knauer armed with a smart line pump 1000 was used, the UV indicator was set at 618 nm, and a UV-visible spectrophotometer (JENWEY, England, model 6405) was used to determinate samples and record the adsorbance of the samples. All adsorbance measurements were performed at 618 nm for the dye using a standard 1 ml optical path quartz cell furnished by Starna (England). The regulation of Labtron pH-meter was performed by a using a Mettler glass electrode PHT-110 [13]. A thermostat bath (Julabo, F12-ED, Germany) that was kept up at the desired hotness was used to achieve the equilibration temperature of the experiments [14].

The article "Adsorption of Malachite Green (MG) as a Cationic Dye on Amberlyst 15, an Ion-Exchange Resin" was published in 2022. Journal: J Environ Public Health.

### 2.2. Reagents and Solutions

The pH of the solutions was adjusted using nitric acid (HNO_3_) and sodium hydroxide (NaOH). Working solutions of MG were made fresh during the day by step-wise dilution of standard existing solutions [15]. All the eluents including acetonitrile, methanol, and water (HPLC grade), and Malachite green powder as oxalate salt were purchased as oxalate salt from a company by the name of Merck in Germany. In this process, the deionized water was obtained from the Millipore Milli-Q filtration method (Bedford, MA, USA). MG existing aqueous solution was prepared and kept in a dark place at 25°C. The specifications of the Amberlyst 15, which was purchased from Sigma, are summed up in Table 1.

### 2.3. Procedure

For the calibration curves, standard working solutions of MG at three concentration levels (1, 5, and 10 mg/l) were tested on different days. The standard curve was plotted to discover the concentration of MG at any time during the period, using the same method as described above.

To investigate the amount of adsorbent, we prepared five malachite green solutions with a concentration of 50 ppm followed by five different packs of the adsorbent with doses of 50, 100, 150, 200, and 250 mg. The MG solutions were added separately to the adsorbent, and the mixtures were stirred for 2 hours. The extraction efficiency in different experiments was calculated as follows:

(1) $$\begin{array}{c} R\left(\%\right)=\left(\frac{C_{0}-C_{t}}{Co}\right)\times 100, \end{array}$$

where *R* represents the percentage of adsorption, *C*_*t*_ is the concentration of MG solution at time *t*, and *C*_0_ is the baseline concentration of MG.

Adsorption capacity (*q*_*t*_) of MG was estimated as follows:

(2) $$\begin{array}{c} q_{t}=\frac{\left(C_{0}-C_{e}\right)\times V}{M}, \end{array}$$

where *q*_*t*_ (mg/g) is the quantity of MG adsorbed onto Amberlyst 15, wet and *C*_0_ and *C*_*e*_ (ppm) are the baseline and balanced concentrations of MG, respectively. *M*(g) represents the molecular weight of MG. *V* represents the volume of the initial solution in liters.

## 3. Results and Discussions

The object of this study is the elimination of malachite green (MG) in the aqueous media, employing the Amberlyst 15, wet, an ion-exchange resin. The tests were conducted to figure out an inexpensive adsorbent for the elimination of malachite green. In this section, the impact of various factors in terms of pH, amount of the adsorbent, concentration of MG, and equilibration temperature on the operational extraction of MG was checked for the purpose of achieving the highest sensitivity. As a final point, the thermodynamic parameters were calculated. The adsorption spectra of MG recorded with Amberlyst 15 wet illuminated the highest adsorption level at 618 nm. Thus, the selected wavelength on which the tests were conducted is 618 nm. The tests were performed by HPLC/UV using an injection volume of 20 *μ*L (Figure 1) and the spectrophotometry method.

The article "Adsorption of Malachite Green (MG) as a Cationic Dye on Amberlyst 15, an Ion-Exchange Resin" was published in 2022. Journal: J Environ Public Health.

### 3.1. pH Impact

We realized that the pH of the solution is a vital factor in the separation process. The impact of the pH on the elimination process on Amberlyst 15, wet with MG, was investigated at the limit of 3–9 by adding nitric acid (HNO_3_) and sodium hydroxide (NaOH). In this situation, MG solution was set at a baseline concentration of 20 mg/L while the temperature and adsorbent dosage were fixed at 25°C and 200 mg, respectively. Dye removal efficiency was enhanced when the pH dropped down from 9 to 3. It comes into sight that an alteration in the pH of the solution leads to diverse ionic sorts. By raising the pH value, the negatively charged surface of the adsorbent and the MG molecules increased. Therefore, the repulsive electrostatic interplays between the adsorbent surface and negatively charged MG increased, leading to a low value of elimination efficiency [16].  Figure 2 illustrated the impact of pH on MG adsorption at 618 nm based on the adsorption capacity (*q*_*e*_ (mg/g)).

At pH values lower than 2 and more than 10, MG gets pale and its adsorbance is decreased [2]. The highest adsorbance is acquired at pH 3.  Figure 3 shows the adsorption of MG as the result of pH. When the pH was increased from 3 to 9, the elimination efficiency was reduced from 88.71 to 65.9%.

### 3.2. Effects of Adsorbent Dosage

The effect of adsorbent dosage on the adsorbance was investigated for 50 mg/L baseline MG concentration by adding various amounts of Amberlyst 15, wet in 100 mL MG solution; other parameters were considered constant.  Figure 4 illustrates the impacts of change in the adsorbent dosage on the function of Amberlyst 15, wet. The elimination efficiency was increased from 79.54% to 99.8% by increasing the adsorbent dosage from 0.05 to 0.25 g. Similar results were obtained in a study conducted by Shirmardi et al., by employing multiwall carbon nanotubes to adsorb reactive dye [17]. The adsorption phenomenon principally is dependent on encountering of the resin and the molecules of the solute [2].

### 3.3. Effects of Primary Concentration of MG on the Elimination Efficiency

The collision time required to attain equilibrium is dependent on the primary MG concentration [18]. The experimental conclusion of adsorptions at miscellaneous concentrations (20, 40, 60, 80, and 100 mg/l of MG) reveals that the MG adsorbed quantity in each unit of resin grew with the increasing concentrations of MG. The equilibrium adsorbent capacity at different levels of MG is shown in Figure 5.

The article "Adsorption of Malachite Green (MG) as a Cationic Dye on Amberlyst 15, an Ion-Exchange Resin" was published in 2022. Journal: J Environ Public Health.

### 3.4. Effects of Temperature

Temperature seems to play a determinant duty in the adsorption procedure; therefore, its results on the adsorption of MG on Amberlyst 15 wet were evaluated. For the effective extraction of phases, we balanced the minimum equilibration time and the least attainable equilibration temperature [12]. The heat can increase the capacity of adsorbance capability. The temperature impact related to effective extraction of MG was thoroughly checked in four courses. This parameter was studied from 15 to 45°C in terms of its impact (Figure 6) and the positive value of Δ*H*° (99.6765 kJ/mol). The adsorbance of MG is an endothermic process because the more we increase the temperature, the better extraction of MG was in terms of effectiveness. Raising the temperature leads to increase in the rate of diffusion of the MG molecules across the external boundary layer and in the internal pores of the adsorbent particles because of the decrease in the viscosity of the solution. According to the results, it is obvious that kinetics methods are relevant to temperature rise, regarding the establishment of equilibrium in shorter interval times through the rise of the temperature [2].

### 3.5. Adsorption Isotherms

This study got some significant information on the surface properties of the adsorbent and its affinity to the adsorbent. The Langmuir model assumes that the uptake of adsorbate molecules occurs without any interaction between adsorbed molecules on a homogenous surface with a finite number of adsorption sites, by monolayer adsorption. When a site is occupied by adsorbate molecules, no further adsorption can occur at that site. The surface will get the saturation point and the maximum adsorption of the surface will be achieved. Langmuir equation that is in the nonlinear form from the previous studies [19, 20] is articulated as follows:

(3) $$\begin{array}{c} q_{e}=\frac{q_{m}bC_{e}}{1+bC_{e}}, \end{array}$$

where *q*_*m*_ represents the highest adsorption capacity in mg/g and *b* is the Langmuir constant in l/mg, which is connected with the power of adsorption joint sites and the surface adsorption energy.

Freundlich isotherm describes the nonideal and reversible adsorption, not restricted to the formation of a monolayer. This model can be applied to multilayer adsorption, with nonuniform distribution of adsorption heat and affinities over the heterogeneous surface. The Freundlich isotherm equation is articulated as follows [21]:

(4) $$\begin{array}{c} q_{e}=K_{f}C_{e}^{1/n}, \end{array}$$

where *K*_*f*_ represents the Freundlich constant connected to the adsorption capacity (mg/g). The larger the value of *K*_*f*_, the higher the adsorption capacity gets. *n* represents the adsorption intensity which is called the heterogeneity coefficient, and the limit rate is from 0 to 1.

The article "Adsorption of Malachite Green (MG) as a Cationic Dye on Amberlyst 15, an Ion-Exchange Resin" was published in 2022. Journal: J Environ Public Health.

The Redlich–Peterson (R–P) isotherm is a three-parameter empirical adsorption model that incorporates elements from both the Langmuir and Freundlich isotherms. The Redlich–Peterson equation is articulated as follows [22]:

(5) $$\begin{array}{c} q_{e}=\frac{AC_{e}}{1+BC_{e}^{g}}, \end{array}$$

where *B* (L/mg) and *A* (L/g) are the Redlich–Peterson empirical coefficients. *g* represents the exponent, and its rate is in the limit of 0 to 1.

Temkin isotherm expresses the decline in the adsorption heat in linear systems instead of logarithmic. At this isotherm, the adsorption energy decreases linearly with the surface coverage due to adsorbent-adsorbate interactions [23]. This is articulated as follows:

(6) $$\begin{array}{c} q_{e}=\frac{\text{RT}}{b_{T}}\ln\left(A_{T}C_{e}\right), \end{array}$$

where *b*_*T*_ represents the Temkin constant relevant to the heat sorption in J/mol, T represents the absolute temperature in K, *A*_*T*_ the Temkin isotherm constant in l/mg, and R the gas constant (8.314 J•mol^−1^•K^−1^).

The conclusions of the adsorption isotherm models were appropriated to Freundlich and Langmuir models (Table 2). The output of our study demonstrated that Redlich–Peterson and Langmuir models describe the data more accurately in Figure 7 and Table 2.

### 3.6. Kinetic Studies

To appraise the adsorption mechanism and its speed control, the fundamental features of a proper adsorbent regarded to adsorption kinetics under optimum solution pH and constant temperature were specified, by using a miscellaneous primary aqueous solution of MG concentrations.

The kinetic statistics posed by pseudo-1st-order (equation (7)) and pseudo-2nd-order (equation (8)) kinetic models are shown in Figure 8 [20, 23].

(7) $$\begin{array}{c} q_{t}=\left(1-\;\exp^{-k_{1}t}\right), \end{array}$$

(8) $$\begin{array}{c} q_{t}=\frac{k_{2}qe^{2}t}{1+k_{2}q_{e}t}, \end{array}$$

where *q*_*e*_ (mmol g^−1^) is the sorption capacity of equilibrium, *t* is the time (min), and *k*_1_ (min^−1^) and *k*_2_ (g mmol^−1^ min^−1^) are the pseudo-1st-order and the pseudo-2nd-order rate constant. The equilibrium sorption capacity, pseudo-1st-order rate constant, and pseudo-2nd-order rate constant were found out tentatively where kinetic models and the slope intercept. If the kinetic model best fits the pseudo-first-order reaction plot by giving *R*^2^ value close to 1, it indicates that the reaction is more inclined towards physisorption. Similarly, if the reaction fits well to pseudo-second-order model, it indicates an inclination toward chemisorption. Several reactions, in general, follow chemisorption initially, and that took over a very short period of time. Kinetic information was found to be in acceptable concurrence with the pseudo-2nd-order kinetics model.

The article "Adsorption of Malachite Green (MG) as a Cationic Dye on Amberlyst 15, an Ion-Exchange Resin" was published in 2022. Journal: J Environ Public Health.

### 3.7. Adsorption Thermodynamics

Adsorption was investigated at various temperatures (15, 25, 35, and 45°C) using 100 ml solution of 100 mg/l of malachite green including 50 mg adsorbent for studying the thermodynamic parameters by the calculation of free energy of Gibbs (DG) as follows[24]:

(9) $$\begin{array}{c} \text{ln}K_{d}=\frac{\Delta S^{{}^{\circ}}}{R}-\frac{\Delta H^{{}^{\circ}}}{RT}, \end{array}$$

where *T*, Δ*S*°, and Δ*H*° are the temperature, entropy, and enthalpy in K, respectively; *R* is the gas constant (8.314 J mol^−1^ K^−1^). The values of entropy (Δ*S*°) and enthalpy (Δ*H*°) are acquired by the intercept of the slope and the ln*K*_*d*_ versus 1 = T plot, which are computed by a curve fitting program [25]. The coefficient of distribution (*K*_*d*_) is computed based on the primary concentration of MG (*C*_*o*_) and the primary concentration of equilibrium of MG in the supernatant (*C*_*e*_) as follows:

(10) $$\begin{array}{c} K_{d}=\frac{C_{o}-C_{e}}{C_{e}}\times \frac{V}{M}, \end{array}$$

where *V* represents the solution volume (mL) and *M* represents the adsorbent mass (g). ∆*G* is the alteration in Gibbs free energy in J mol^−1^, computed as follows [24]:

(11) $$\begin{array}{c} \Delta G^{{}^{\circ}}=\Delta H^{{}^{\circ}}T-\Delta S^{{}^{\circ}}. \end{array}$$

The impact of temperature on MG adsorption on Amberlyst 15 wet has been demonstrated by a linear plot of ln*K*_*d*_ versus 1/T in Figure 9, and the calculated thermodynamic parameters and correlation coefficients are computed from equations (9) and (11) are abridged in Table 3. The positive value of Δ*S*° (333.1253 J/K mol) gives back randomness at the solid-liquid interface all the while sorption.

## 4. Conclusion

Amberlyst 15 wet was successfully employed for the sake of removal of dangerous dye malachite green. A brief report on the performance of some other adsorbents is summarized in Table 4. The results indicate that the Amberlyst 15 wet resin could be considered an acceptable alternative for drawing out the dye from aqueous solutions. Compared to the other adsorbents for malachite green removal procedure, this method takes place in a shorter period of time. With regard to the thermodynamic data obtained, adsorption of the dye by Amberlyst 15 emerged to be a physical mode and this is an endothermic and spontaneous process. The positive value of Δ*S*° demonstrates randomness at the solid-liquid interface of sorption. According to the results, it is a cost-effective and efficient adsorbance method, compared with many other toxic substance removal processes from aqueous environments.

The article "Adsorption of Malachite Green (MG) as a Cationic Dye on Amberlyst 15, an Ion-Exchange Resin" was published in 2022. Journal: J Environ Public Health.

## Figures and Tables

**Figure 1:** The chromatograms. The samples were spiked with 5 and 0.5 *μ*g/L of malachite green, respectively. The retention time of malachite green was 3.55 min. The detector-monitoring wavelength was 618 nm.

**Figure 2:** The results of pH effects on the adsorption of 20 mgL^−1^ of malachite green (MG) dye with 200 mg Amberlyst 15 wet in 100 ml solution based on the adsorption capacity (*q*_*e*_ (mg/g)).

**Figure 3:** The effect of pH on the adsorption percent of 20 mgL^−1^ of malachite green (MG) with 200 mg Amberlyst 15 wet in 100 ml solution.

**Figure 4:** The effect of Amberlyst 15 wet concentration on the adsorption of 50 ppm of malachite green (MG) in 100 ml dye solution.

**Figure 5:** Effect of initial concentration of MG on the removal efficiency.

**Figure 6:** Temperature impact on the extraction of 100 ml of malachite green (MG) solution, 100 ppm (in the presence of 50 mg adsorbent, encounter time of 4 hours, and pH 3).

**Figure 7:** Adsorption isotherm of MG on Amberlyst 15 wet at initial malachite green (MG) concentration from 20 to 100 mg/l, adsorbent dosage of 100 mg, pH 3.0, and 25°C for 220 mins.

**Figure 8:** Pseudo-second-order and pseudo-first-order kinetic models of malachite green (MG) adsorption on Amberlyst 15 wet (in the presence of 100 mg adsorbent, contact time of 220 min, and pH 3).

**Figure 9:** Plots of ln*K*_*d*_ versus 1/T for malachite green (MG) adsorption on Amberlyst 15 wet at the adsorbent dose of 400 mg/l, pH 3.0, and different temperatures.

**Table 1:** Main properties of Amberlyst 15 wet used in the present study.

Parameter	Specifications
Appearance	Brown-grey beads
Molecular formula	C_18_H_18_O_3_S
Density	0.75
Ionic form as shipped	H+
Concentration of acid sites^‡^	≥4.70 eq/kg
Catalyst volatiles	≤1.6%
Water solubility	Insoluble in water
Sensitivity	Hygroscopic
Total volume capacity	>1.70 eq/l
Total weight capacity	>4.70 eq/kg
Moisture retention capacity	52.0 to 57.0%
Mean particle size	0.600 to 0.850 mm
Uniformity coefficient	<1.70
Particle density	1.70 g/mL
Water content	52–57%

**Table 2:** Langmuir and Frendlich, Redlich–Peterson, and Temkin parameters of MG adsorption on Amberlyst 15 wet.

Models	Parameters			
Langmuir	*q*_*m*_, mg/g	*b*, L/mg	*R* ^*2*^	
	46.58	1.463	0.9880	

Freundlich	*K*_*F*,_ (mg/g) (L/mg)^1/n^	*N*	*R* ^*2*^	
	28.25	7.40	0.9360	

Redlich–Peterson (R–P)	*A*, L/g	*B*, L/mg	*γ*	*R* ^*2*^
	55.41	1.004	1.049	0.9933

Temkin	*b*_*T*_, J/mol	*A*_*T*_, L/mg	*R* ^2^	
	474.36	193.23	0.9490	

The article "Adsorption of Malachite Green (MG) as a Cationic Dye on Amberlyst 15, an Ion-Exchange Resin" was published in 2022. Journal: J Environ Public Health.

**Table 3:** Thermodynamic parameters malachite green (MG) adsorption on Amberlyst 15 wet at different temperatures in Kelvin (initial concentration of MG is 100 mg/L).

Δ*H*° (kJ/mol)	Δ*S*° (J/mol K)	Δ*G*° (kJ/mol)				*R*_2_
		288°K	298 K	308°K	318 K	
99.6765	333.1253	3.7364	0.4051	−2.92606	−6.2573	0.9616

**Table 4:** Comparison of the maximum adsorption of MG onto various adsorbents.

Adsorbent	*R* (mg/lit)	Reference
Modified *γ*-alumina	91.61%	[26]
Phytogenic magnetic nanoparticles	98.57%	[27]
Activated carbon of catha edulis stem	83.65%	[28]
Extracellular polymeric substance of *Lysinibacillus* sp.SS1	99.01 ± 0.61%	[29]
Amberlyst 15 an ion exchange resin	98.27%	This study

## Data Availability

Upon request, the data supporting the conclusion of our study are accessible from the corresponding author.
